The article "Cardioprotective activity of placental growth factor in a rat model of acute myocardial infarction: nanoparticle-based delivery versus direct myocardial injection" was retracted in 2015. Reasons: compromised peer review; ethical violations by an institution or third party; concerns about a third party's involvement.

# Cardioprotective activity of placental growth factor in a rat model of acute myocardial infarction: nanoparticle-based delivery versus direct myocardial injection

**DOI:** 10.1186/1471-2261-14-53

**Published:** 2014-04-17

**Authors:** Zhe-xin Lu, Li-li Mao, Feng Lian, Jun He, Wen-tian Zhang, Chen-yang Dai, Song Xue, Wei-gen Lu, Hong-sheng Zhu

**Affiliations:** 1 Department of Cardiovascular Surgery, Ren Ji Hospital, School of Medicine, Shanghai Jiao Tong University, 160 Pu-Jian Rd, Shanghai 200127, People’s Republic of China; 2 National Pharmaceutical Engineering Research Center, China State Institute of Pharmaceutical Industry, 1111 Zhong-shan North 1 Rd, Shanghai 200437, People’s Republic of China

**Keywords:** Placental growth factor, Acute myocardial infarction, Cardiac function, Nanoparticles-mediated drug delivery, Vicious ventricular remodeling

## Abstract

**Background:**

To comparatively evaluate the cardioprotective activity of placental growth factor (PGF) delivered through direct injection and a nanoparticle-based system respectively and to study the underlying mechanisms in a rat model of acute myocardial infarction (AMI).

**Methods:**

Poly lactic-co-glycolic acid (PLGA)-based PGF-carrying nanoparticles (PGF-PLGA_NPs_) were created. The mean size and morphology of particles were analyzed with particle size analyzer and transmission electronic microscopy (TEM). Encapsulation efficiency and sustained-release dose curve were analyzed by ELISA. Sprague-Dawley rats were randomized into four groups (n = 10). While animals in the first group were left untreated as controls, those in the other 3 groups underwent surgical induction of AMI, followed by treatment with physiological saline, PGF, and PGF-PLGA_NPs_, respectively. Cardiac function was evaluated by transthoracic echocardiography at 4 weeks after treatment. At 6 weeks, rats were sacrificed, infarction size was analyzed with Masson trichrome staining, and protein contents of TIMP-2, MT1-MMP and MMP-2 at the infarction border were determined by immunohistochemistry and western blotting analysis.

**Results:**

PGF was released for at least 15 days, showing successful preparation of PGF-PLGA_NPs_. Coronary artery ligation successfully induced AMI. Compared to physiological saline control, PGF, injected to the myocardium either as a nude molecule or in a form of nanoparticles, significantly reduced infarction size, improved cardiac function, and elevated myocardial expression of TIMP-2, MT1-MMP, and MMP-2 (P < 0.05). The effect of PGF-PLGA_NPs_ was more pronounced than that of non-encapsulated PGF (P < 0.05).

**Conclusion:**

Target PGF delivery to myocardium may improve cardiac function after AMI in rats. PLGA-based nanoparticles appear to be a better approach to delivery PGF. PGF exerts its cardioprotective effect at least partially through regulating metalloproteinase-mediated myocardial tissue remodeling.

## Background

Paracrine factors derived from stem cells have been demonstrated to be capable of improving cardiac function after myocardial infarction (MI) and are now becoming a hot topic of myocardial regeneration research [1,2]. One of these factors is placental growth factor (PGF). A beneficial role for PGF in heart failure has been previously demonstrated in an animal study where autoimplantation of myoblasts overexpressing PGF into myocardium resulted in a significant functional improvement in the failing heart after ischemic MI [3]. However, the mechanisms underlying the benefits of PGF in MI-associated heart failure have yet to be further elucidated.

It has been documented that MI results in remodeling of the myocardium, including the extracellular matrix (ECM) [4]. Tissue inhibitors of metalloproteinases (TIMPs) are critical regulators of ECM integrity, capable of inhibiting the activity of ECM-degrading enzymes, matrix metalloproteinases (MMPs) [5]. Numerous types of MMPs have been identified in mammals, of which membrane-type-I MMP (MT1-MMP) is of a particular importance in the regulation of ECM integrity. Through activating MMP-2, MT1-MMP may aggravate the degradation and loss of ECM [6]. However, it remains unclear whether PGF may exerts its beneficial effect against ischemic myocardial injury through regulating MMP-dependent ECM degradation in the myocardium.

Various approaches to delivery exogenous agents including PGF have been developed, of which, nanoparticles have attracted considerable attention in recent years worldwide [7]. Poly (lactic-co-glycolic acid) (PLGA), a biodegradable polymer approved by U.S. Food and Drug Administration for drug delivery, is one of the widely used types of carriers [8]. Due to its properties of surface erosion and subsequent constant matrix erosion, PLGA allows for slow drug release [9]. Besides sustained release, PLGA-based nanoparticles as drug carriers possess advantages of increased freedom and better permeability into interstitial spaces. Nevertheless, delivery of PGF-carrying PLGA nanoparticles (PGF-PLGA_NPs_) into myocardium has been seldom reported.

This study aimed to investigate the therapeutic efficacy of PGF-PLGA_NPs_-bearing nanoparticles against acute myocardial infarction (AMI) in comparison with direct administration of PGF as well as the mechanistic role of TIMP-2, MT1-MMP and MMP-2-regulated cardiac remodeling in PGF-mediated cardioprotection in a rat model.

## Methods

All human studies have been approved by shanghai Ren Ji Hospital Ethics Committee and performed in accordance with the ethical standards

### Preparation of PGF-PLGA_NPs_

PLGA (100 mg; block ratio: 50:50; viscosity: 0.53 dl/g; average molecular weight: 6.0 × 10^4^), purchased from Shandong Institute of Medical Devices (Shandong, China), was dissolved in 0.5 ml ethyl acetate as an oil phase (O). Recombinant human PGF, purchased from R&D Systems (catalog #264-PG-050, Minneapolis, MN, USA), was dissolved in H_2_O (0.50 μg/μl) as a water phase (W1). W1 was then dripped slowly into O to create the W1/O emulsion through ultrasonication. W1/O was added into 2 ml 19% pluronic F-68 solution to form W1/O/W2 double emulsions. Ethyl acetate was evaporated under a vacuum and the PLGA nanoparticles were collected after high speed centrifugation (6000 rpm, 8 min). Finally, PGF-PLGA_NPs_ were lyophilized. The dose of PGF was chosen based on a previous study [10].

### Assessment of *in vitro* release kinetics and encapsulation efficiency

To analyze *in vitro* release kinetics, PGF-PLGA_NPs_ (containing 30 μg PGF) were suspended in 16 ml of phosphate-buffered saline (PBS, PH 7.4). The suspension solution was then placed in an environment of 37°C with horizontal shaking for 15 days. During this period, 1 ml of the medium was sampled twice (12 h and 24 h) on the first day and once every two days thereafter. The concentration of PGF released at different time points was determined by enzyme-linked immunosorbent assay (ELISA) as previously described [11]. All experiments were conducted in triplicate. The amount of encapsulated PGF was determined as the difference between the initial amount and residual amount in the supernatant. The average size and morphology of the nanoparticles were assessed under the NICOMP380 ZLS (Particle sizing systems, USA) and H-600 transmission electron microscopy (HITACHI, Japan). The percent encapsulation efficiency was calculated as: $=\frac{\left(\mathrm{Mass}\;\mathrm{of}\;\mathrm{total}\;\mathrm{drug}‒\mathrm{Mass}\;\mathrm{of}\;\mathrm{free}\;\mathrm{drug}\right)}{\mathrm{Mass}\;\mathrm{of}\;\mathrm{total}\;\mathrm{drug}}\times 100\%$, and the drug loading as:

$$=\frac{\left(\mathrm{Mass}\;\mathrm{of}\;\mathrm{total}\;\mathrm{drug}‒\mathrm{Mass}\;\mathrm{of}\;\mathrm{free}\;\mathrm{drug}\right)}{\mathrm{Mass}\;\mathrm{of}\;\mathrm{microspheres}}\times 100\mathrm{\%.}$$

### Animals, AMI induction and treatment

Sprague-Dawley rats (250 ± 50 g, 8-10 weeks) were obtained from the Experimental Animal Center, Shanghai Jiaotong University-Affiliated Renji Hospital, China. They were housed in groups (4 per cage) with free access to a regular diet and clean drinking water. All the experimental procedures described below adhered strictly to the guidelines set forth by the National Science and Technology Commission of China and approved by the institutional ethics committee.

For AMI induction, rats were anesthetized with an intraperitoneal dose of 0.2 ml 2% pentobarbital under intubated mechanical ventilation at 80 breaths per minute. Thoracotomy was performed through the fourth intercostal space, and the left anterior descending coronary artery was identified and ligated with 6.0 prolene suture in the middle portion. A few minutes after ligation, pallor and akinesia were seen in the anterior wall and apical left ventricular area. The interface between the pale and normal areas was defined as ‘infarction border zone’. The presence of infarction zone and ST segment elevation were considered as criteria of successful induction of AMI. A group of animals (n = 10) were left untreated controls. The animals that were successfully induced to develop AMI were randomized to receive 30 μl PBS (n = 10), non-encapsulated PGF (2 μg in 30 μl solution, n = 10), and PGF-PLGA_NPs_ (2 μg in 30 μl solution, n = 10), respectively. The injection of 30 μl was administrated around the pale areas: upper, center, and lower with 10 μl in each area. All agents were delivered to the infarction border zone through intramyocardial injection using a micro-syringe.

### Cardiac function determination

Echocardiographic examinations were performed 4 weeks after surgery under inhaled isoflurane (0.2%) anesthesia, with the Vevo770 ultrasound system (Visualsonics Inc., Toronto, Canada). The frequency of the probe was set at 17.5 MHz, sampling frequency in M-mode at 1000/s, and scanning speed 50-100 mm/s. The probes were placed on precordium and the detection was carried out from the section of ventricular bands. Left ventricular anterior wall (LVAW) thickness, left ventricular end-diastolic diameters (LVEDD), and left ventricular end-systolic diameters (LVESD) were measured. Based on these measurements, left ventricular end-diastolic volume (LVEDV), left ventricular end-systolic volume (LVESV), left ventricular ejection fraction (LVEF) and left ventricular fraction shortening (LVFS) were calculated as follows:

$$\begin{array}{l} \mathrm{LVEDV}=\frac{7.0\times {\mathrm{LVEDD}}^{3}}{\left(2.4+\mathrm{LVEDD}\right);}\\ \mathrm{LVESV}=\frac{7.0\times {\mathrm{LVESD}}^{3}}{\left(2.4+\mathrm{LVESD}\right);}\\ \mathrm{LVEF}=\frac{\left(\mathrm{LVEDV}‒\mathrm{LVESV}\right)}{\mathrm{LVEDV}}\times 100\%;\\ \mathrm{LVFS}=\frac{\left(\mathrm{LVEDD}‒\mathrm{LVESD}\right)}{\mathrm{LVEDD}}\times 100\%. \end{array}$$

### Scar area analysis

Six weeks after AMI surgery, rats were anesthetized by inhaled isoflurane (0.2%) followed by cardiac perfusion with 100 ml 4% triformol. Animals were then sacrificed by rapid excision of heart. Hearts were excised and soaked immediately in saline to remove the excess blood from the ventricles before being fixed in 4% triformol. Paraffin-embedded samples were sectioned at 5 μm and Masson’s trichrome staining was performed. Digital images of the stained sections were captured and tissue scar was analyzed with Image Pro-Plus 6.0 software. The size of infarct was also calculated as previously described [12].

### Imunohistochemical analysis

This was performed using the DAKO EnVision™ + System (Glostrup, Denmark). Briefly, paraffin-embedded sections (5 μm) were dewaxed, and incubated with the primary antibody TIMP-2 (Abcam, Cambridge, MA, USA, catalog #ab1828), MT1-MMP (Abcam, catalog #ab51074), MMP-2 (Abcam, catalog # ab80737) and Envision. After the visualization with diaminobenzidine (DAB), images were acquired under the Axioplan 2 automatic fluorescence microscopy (Carl Zeiss) and the intensity of the corresponding protein bands were analyzed using the Axioplan 2 imaging software.

### Western blotting analysis

Infarcted tissue specimens collected from the border zone were homogenized in 1% Triton X-100, 10 mM Tris-HCl (PH 7.6). After centrifugation at xxxx g for xx min, the supernatant was collected. Concentration of total proteins in the supernatant was quantitated. Ten μg proteins from each sample prepared in a buffer containing 2% sodium dodecyl sulfate (SDS) were separated by electrophoresis on a SDS-PAGE and then transferred to a nitrocellulose membrane blot. After blocking in 5% skimmed milk in TBST (0.1% Tween 20) for 1 hour, the blot was incubated with primary antibodies respectively against TIMP-2 (Abcam, ab1828), MT1-MMP (Abcam, ab51074), MMP-2 (Abcam, ab80737) at 4°C overnight. Following washing, the blot was incubated with a HRP anti-rabbit secondary antibody (Santa Crutz, CA, USA) for 1 hour at room temperature. After another three rounds (10 min/time) of washing in TBST, the blot was developed by enhanced chemiluminescence (ECL) as instructed by the manufacturer. For the purpose of loading control, the blot was stripped and re-probed with GAPDH. The immunoreactive bands of the interest protein and GAPDH protein were densitometricaly analyzed with Image J software (National Institutes of Health, USA).

### Statistical analysis

Data were expressed as mean ± standard deviation. Intergroup comparison was analyzed by t test, and the intra comparison was conducted by paired t test. All statistical analyses were performed using SPSS 10.7 software (Chicago, IL, USA). Differences were considered significant when P < 0.05.

## Results

### Characterization of PGF-PLGA_NPs_

PGF-PGF-PLGA_NPs_ had a regular spherical shape with good integrity, even distribution, and smooth surface, as demonstrated by electron microscopy (Figure 1A). The average diameter of the nanoparticles was 233.9 ± 15.3 nm and the average encapsulation efficiency was 43.52 ± 4.21% (Figure 1B).

**Figure 1:** **Characterization of nanoparticles. A**: morphology revealed by transmission microscopy. **B**: bar graphs, showing the average diameters detected by NICOMP 380 ZLS.

### *In vitro* release kinetics of PGF-PLGA_NPs_

Shown in Figure 2 are concentrations of PGF released from PGF-PLGA_NPs_ at different time points during the 15-day experiment as determined by ELISA. In the first 1-5 days, PGF release was rapid, amounting for more than 60% of the total release. After that, the daily release amount became more stable. By day 14 or 15, 80% of PGF was released.

**Figure 2:** ***In vitro *** **cumulative release curve of PGF-PLGA**_**NPs **_**nanoparticles.**

### Echocardiography findings

Echocardiography was performed on all animals at 4 weeks after surgery. Compared to animals in the sham group (Figure 3A), those in the other three groups showed different degrees of enhanced myocardial echo, thinning of the left ventricular wall and weakened contractions (Figure 3B-D). The LVEF, LVFS, and LVAW in PGF-PLGA_NPs_ group were all significantly higher than those in the PGF and AMI control groups (P < 0.05, Table 1).

**Figure 3:** **Echocardiography of rats in the control group (A), AMI group (B), PGF group (C) and PGF-PLGA**_**NPs **_**group (D) at the end of the fourth week after AMI surgery.**

**Table 1:** Cardiac function parameters assessed by echocardiography

	**Parameters**			
**Groups**	**LVEF (%)**	**LVFS (%)**	**LVAW (mm)**	**Heart rate**
Sham	81.28 ± 3.70	51.78 ± 11.26	3.23 ± 0.60	478 ± 47
AMI	21.03 ± 6.36^#^	8.74 ± 4.08^#^	0.87 ± 0.14^#^	497 ± 52
PGF	27.71 ± 4.59^#^&	16.29 ± 6.91^#^&	1.28 ± 0.28^#^&	462 ± 61
PGF-PLGA_NPs_	40.61 ± 8.11^#^&^※^	26.63 ± 9.27^#^&^※^	1.35 ± 0.38^#^&	481 ± 59

*AMI* acute myocardial infarction; *LVEF* left ventricular ejection fraction; *LVFS* left ventricular fraction shortening; *LVAW* Left ventricular anterior wall. ^#^p < 0.05, compared with sham group; & p < 0.05, compared with AMI group; ^※^p < 0.05, compared with PGF group.

### Myocardial scar

Shown in Figure 4 are Masson trichrome staining results. There were significant differences (P < 0.05) in the average scar area between groups (Figure 4A). In the cardiac tissue sections, viable myocardium was stained red, while fibrosis due to infarction damage was stained blue. In the sham operation control group, no area was stained blue (Figure 4B1). In contrast, the infarcted zone in the non-treatment AMI control group was filled with blue scar tissues (Figure 4B2). Treatment with both non-encapsulated PGF (Figure 4B3) and PGF-PLGA_NPs_ (Figure 4B4) reduced the area stained blue and the intensity of blue staining. However, the effect of PGF-PLGA_NPs_ was more pronounced; myocardial compensatory hypertrophy was seen in the PGF group.

**Figure 4:** **Effect of PGF on myocardial scar formation after AMI. A**: A bar graph showing the average scar area in different groups. Symbols indicate significant differences (P < 0.05) from the control group (^#^), from the non-treatment AMI group (&), and from the nude PGF group (^※^), respectively. **B**: Digital images (×7.5) of tissue sections stained by Masson Trichrome in the control group **(B1)**, AMI group **(B2)**, PGF group **(B3)** and PGF-PLGA_NPs_ group **(B4)**. Red color indicates viable myocardium, while blue color indicates fibrosis due to infarction damage.

### Protein contents of TIMP-2, MT1-MMP, and MMP-2

Shown in Figure 5 are the results of immunohistochemical staining assessment of TIMP-2, MT1-MMP, and MMP-2 protein signals in the cardiac specimens (Figure 5). The immunoreactive signal for TIMP-2 was strong in the sham operation group but became significantly weakened after AMI surgery (P < 0.05). Both non-encapsulated PGF and PGF-PLGA_NPs_ significantly attenuated AMI-associated decrease in the reactive signal for TIMP-2 (P < 0.05). In contrast, immunoreactive signals for MT1-MMP and MMP-2 all showed a pattern of changes in different groups totally opposite to the pattern for TIMP-2.

**Figure 5:** **Immunohistochemical signals of TIMP-2 (A1-D1), MT1-MMP (A2-D2), and MMP-2 (A3-D3) (×200) in myocardium in the control group (A), non-treatment AMI group (B), PGF group (C), and PGF-PLGA**_**NPs **_**group (D).** The densitometric data on the corresponding signals in **A**, **B**, **C** and **D** are presented as bar graphs in **E**. Symbols indicate significant differences (P < 0.05) from the control group (^#^), from the non-treatment AMI group (&), and from the nude PGF group (^※^), respectively.

Changes in TIMP-2, MT1-MMP, and MMP-2 protein contents in different groups were also analyzed by Western blotting. Similar patterns to those for these proteins shown in immunohistochemical staining were observed (Figure 6).

**Figure 6:** **Content changes of TIMP-2, MT1-MMP, and MMP-2 detected by western blotting. A**: Representative Western blots, showing bands of TIM-2, MT1-MMP and MMP-2 in myocardial specimens collected from the indicated groups. **B**: Bar graphs, showing the densitometric data corresponding to **A**. Symbols indicate significant differences (P < 0.05) from the control group (^#^), from the non-treatment AMI group (&), and from the nude PGF group (^※^), respectively.

## Discussion

MI is a life-threatening clinical condition. Even though the symptoms of myocardial ischemia can be partly improved by pharmacologic agents, delivered either surgically or non-surgically, yet the malignant myocardial remodeling caused by MI cannot be reversed. PGF, one of the cytokines belonging to VEGF family, binds to flt-1 receptors in its target cells including cardiac myocytes, cardiac fibroblasts, and bone marrow derived cells [13] and then activates downstream signals important in myocardial damage repair [14,15], angiogenesis [16], inflammatory response [17], and peripheral stem cell distribution [18]. Given that PGF intervention after AMI results in an increase in specific gene transcripts, PGF is regarded as a prognostic marker of acute coronary syndrome [19]. To evaluate the cardioprotective potential of PGF, we determined the effect of PGF, injected into the infarction zone of the myocardium either as a nude molecule or in a form of nanoparticles, on the cardiac function after AMI in a rat model in this study. First, we found that both PGF and PGF-PLGA_NPs_ significantly increased LVEF, reduced scar tissue formation, thus leading to recovery of cardiac function, in animals after AMI induction. However, the improvement in all these variables was more significant for PGF-PLGA_NPs_ than PGF.

In order to investigate the mechanism underlying the cardioprotective activity of PGF, we analyzed changes in protein contents of MMPs (MT1-MMP, MMP-2) and its inhibitor (TIMP-2) in infarcted area. The protein content of TIMP-2 at the baseline level was high, but it was reduced after-AMI. PGF intervention was effective to attenuate the reduction. In contrast, an opposite pattern of changes was observed for MT1-MMP and MMP-2 proteins. MMPs belong to a family of Zn^2+-^dependent enzymes known to cleave ECM proteins under normal and pathological conditions [20,21]. TIMP-2 may promote the conversion from pro-MMP-2 to mature MMP-2, acting as a key protein regulating ECM degradation after AMI [22]. Under exogenous PGF intervention, a compensatory increase in TIMP-2 and MT1-MMP expression occurs, leading to an increased production and/or activation of pro-MMP-2 through MT1-MMP [23]. In the process of ECM degradation, MT1-MMP and MMP-2 exert synergistic effects; type I collagen is initially degraded by MT1-MMP and the product subsequently degraded by MMP-2 [23,24]. Our observations in this study are consistent with the established cascade of ECM degradation in the infarcted myocardial zone after AMI. We also observed myocardial necrosis and collagen, followed by gradual scarring. A large area of blue scar tissues was detected in AMI group, followed by a decrease in TIMP-2 protein content in the myocardium. Following PGF intervention, both TIMP-2 and MMP-2 increased in protein content, resulting in accelerated collagen degradation, in the scar tissue in the MI zone, facilitating the implantation of the new-born cardiomyocytes. TIMP-2 is a natural inhibitor of both MT1-MMP and MMP-2. TIMP-2 deficiency completely abrogates MMP-2 activation but markedly increases activities of various collagenases, particularly MT1-MMP , after MI [5]. Based on our immunohistochemical and Western blotting analysis results, we suggest that post-AMI intervention with PGF may promote the expression recovery of TIMP-2, thus activating MMPs, inhibiting the formation of scar tissues and improving ventricular remodeling.

Nanoparticles are submicron-sized polymeric particles encapsulated with a therapeutic agent within the polymeric matrix or conjugated or absorbed onto their surface [25], allowing for a controlled release of active agents to the specific site of action at a therapeutically optimal rate [26]. PGF has a short half-life and is not suitable to be exposed in tissues. To obtain a sustained slow-release, multiple types of the nanoparticles have been used to deliver PGF in human body. For instance, in the study of Mohammed et al, they used chitosan-alginate nanoparticle [10], while in this study PLGA was used. We showed that nanoparticles-based delivery enabled persistent and sustained release of PGF, supporting the superiority of nano-materials in drug delivery [27], due to their excellent biocompatibility and biodegradability [28]. It was consistent with the study of Mohammed et al. and others [29,30]. The main advantage of using PLGA as a carrier is that the release profile can be modified by different parameters, such as molecular weight and lactide to glycolide ratio. In this study, a consistently slow release of PGF from nanoparticles was demonstrated during the 15-day period of test. Another advantage of PLGA-based drug delivery is a burst release in the initial period. In this study, an initial burst release of PGF (10% of total approximately) was observed on the first day. Given significant increases in the expression of pro-inflammatory cytokines and MMPs the first 3 days after AMI [31], the burst release of PGF observed in this study may have important clinical implications.

## Conclusion

PGF may improve the cardiac function after AMI, possibly through a mechanism involving TIMP-2, MT1-MMP, and MMP-2-associated ECM degradation ad tissue remodeling in the myocardium. Due to well-controlled release properties, PGF-PLGA_NPs_ system developed in this study offers a superior approach of myocardial delivery of PGF. Further studies are warranted on the mechanisms underlying the cardioprotective activity of PGF in AMI as well as on the optimized dose and administration time window of PGF-PLGA_NPs_ as a potential therapeutic approach for AMI.

## Competing interests

The authors declare that they have no competing interests.

## Authors’ contributions

ZXL and LLM carried out the molecular genetic studies, participated in the sequence alignment and manuscript preparation. FH and JH carried out the immunoassays. WTZ participated in the sequence alignment. CYD, SX and WGL participated in the design of the study and performed the statistical analysis. HSZ conceptualized the study, participated in the study design, oversaw execution of the designed experiments and helped prepare the manuscript. All authors read and approved the final manuscript.

## Authors’ information

Zhe-xin Lu and Li-li Mao should be regarded as co-first authors.

## Pre-publication history

The pre-publication history for this paper can be accessed here:

http://www.biomedcentral.com/1471-2261/14/53/prepub

## Fundings

Shanghai Education Commission (11YZ48), Shanghai Education Commission (13ZZ091), Shanghai municipal Scientific & Technological Commission (12 nm0502100), Shanghai Municipal Bureau of Health P.R. China (No.20114243)
